# High-Performance Computing Analysis and Location Selection of Logistics Distribution Center Space Based on Whale Optimization Algorithm

**DOI:** 10.1155/2022/2055241

**Published:** 2022-06-22

**Authors:** Lijuan Yang, Xiedong Song

**Affiliations:** ^1^School of Management, Anhui Business and Technology College, Hefei 231131, China; ^2^School of Intelligent Engineering, Yantai Institute of Science and Technology, Yantai 265600, China

## Abstract

As a meta-heuristic algorithm based on swarm intelligence, the WOA algorithm has few control parameters and searches for the optimal solution by encircling the prey, searching for the prey, and attacking the bubble net. During the whole process, only two internal parameters A and C are utilized for the control of the exploration and development process. BWOA is simple to implement. In the process of algorithm execution, the initial population, global exploration, and local development stages have shortcomings. Therefore, it is necessary to optimize the WOA algorithm. Based on WOA, this study conducts a high-performance computing analysis and location selection of logistics distribution center space. It is concluded that: (1) by using the combination of direct logistics distribution and hierarchical logistics distribution, the WOA algorithm optimizes the cross selection strategy, the population fitness S-LO is improved, the quality of LA is guaranteed, and the chaotic S-LO mapping eliminates inferior individuals in the population. Direct distribution is carried out for bulky goods and important distribution customers, and hierarchical logistics distribution is used for customers in intensive logistics distribution destinations. (2) WOA uses the second reverse learning, chaotic mapping, and logistic chaotic mapping to improve the location update mode. The direct distribution method is mostly used for the logistics business with short journeys, fixed distribution points, and more goods delivered at one time, and logistics enterprises do not need to store and distribute goods. The uniform ergodicity of the Tent chaotic map and logistic chaotic map is improved. Ka adaptive inertia weights are a good complement to optimize the limitations of the Ao whale algorithm. (3) The inertia weight of the levy flight behavior can play a powerful role in balancing the global exploration ability and optimization performance of the intelligent algorithm. The long-term short-distance search of HED and the long-distance jump of KVAR are combined. Variant individuals undergo vector synthesis. It reduces the construction and operation costs of logistics sites and is suitable for logistics distribution under specific conditions.

## 1. Introduction

Whale Optimization Algorithm (WOA), as a new type of modern intelligent optimization algorithm, has been applied in research fields such as reactive power scheduling optimization, short-term load forecasting, logistics distribution calculation analysis, and location selection and has shown good results. Head whales surround the fish in a circular contraction [1–3]. At the same time, it will swim upward in a spiral upward manner to prey, and by following a “9” or “O”-shaped path, it is constantly approaching its prey while generating unique bubbles. The position of each humpback whale in the whale algorithm represents a feasible solution. The advantages of this algorithm are that there are few adjustment parameters, simple operation, and strong local optimal ability. For each basic function, define the population size and variable range, run the improved whale optimization algorithm 30 times from randomly generated different populations, and calculate the average and standard deviation as the basis for judging the optimization effect of the algorithm. In the whale algorithm, each whale can be regarded as a particle, and the position of each particle represents a decision variable. The shrinkage and encirclement mechanism will make the remaining whale individuals move closer to the current optimal whale, and the change in the absolute value of the coefficient will affect the judgment of the remaining whales based on the current position of the corresponding position of the optimal position at the next moment. The spiral update mechanism is based on the distance between the whale's real-time position and the current optimal position, simulating the whale's predation through a spiral trajectory to explore the trajectory range. This makes the population develop towards a single, prone to premature convergence. The optimal individual is mutated [4]. Individuals with high fitness before and after mutation can be used to expand the search range and improve population diversity [5–7]. The core idea of the WOA algorithm is to abstract the hunting mode of humpback whales into a mathematical model, which subtly solves the problem of finding the optimal value in most scenarios, but when faced with some more complex problems or high search space dimensions, in the WOA algorithm, there is insufficient global exploration ability and unsatisfactory convergence accuracy. It is easy to fall into problems such as local optimum [8–10]. In the process of algorithm execution, the initial population, global exploration, and local development stages have shortcomings. For the meta-heuristic algorithm based on group iteration, the quality of the initial population will directly affect the optimization ability and stability of the algorithm and the high-quality initial population with better diversity can lay the foundation for the global search of the group iterative algorithm. Since there is no prior knowledge of the global optimal value of the problem to be solved, the WOA algorithm uses random initialization to generate the initial whale population. The initialized population generated by the random method cannot guarantee the diversity of the population, and it is difficult to effectively extract the useful information of the solution space. To a certain extent, it will affect the convergence speed and optimization ability of the algorithm. The location update of whale individuals in the global exploration phase mainly depends on two parts: the randomly selected search individual location and the product of the coefficient vectors A and D. In the iterative process, A decreases from 2 to 0 and the proportion of A greater than 1 is very small, which leads to a very low probability of global exploration of the whale population, which further weakens the global exploration ability, and it is difficult to get rid of the constraints of local optimality, which leads to the algorithm Precocious and convergent.

As a key node in the express distribution process, logistics distribution sites have received more and more attention. Successful distribution site selection can speed up the circulation efficiency of products and reduce logistics costs, bringing convenience and economic benefits to suppliers and demanders. The development of social productive forces is promoted. Logistics and distribution need to deliver goods from suppliers to customers. For customers, logistics and transportation efficiency is an important determinants of customer experience. In the process of logistics and transportation, storage, transportation, distribution, and processing are all indispensable. In the process of applying the whale algorithm to solve the optimization problem, since the convergence ability of the algorithm is closely related to the size and randomness of the population, the reasonable setting of the population is very important to the subsequent operation of the algorithm. The differential evolution algorithm performs mutation operations according to the differential strategy. The most prominent feature of the algorithm is its mutation operator. The method of selecting the parent in the mutation operator has an important impact on the search speed of the optimal solution of the differential evolution algorithm. Reasonable allocation of resources is suitable for demand distribution. It also needs to adapt to the overall function and spatial distribution pattern of the city [11–13]. Huge investment, recovery, and relocation are all difficult. The infrastructure of the logistics distribution center is coordinated and balanced with the overall logistics system in terms of spatial distribution, productivity, and technical capabilities. To control the impact of site selection on urban traffic is tried [14, 15]. The whale optimization algorithm has the characteristics of simple structure and easy implementation, but there is a problem of local optimality. It can be improved by simulating the mutation and selection operation of the differential evolution algorithm, so that the improved algorithm not only has the ability to quickly converge but also can optimize globally.

## 2. Logistics Model

### 2.1. Enterprise Logistics Distribution Network Model

The multilevel network distribution method is generally used in the logistics network distribution of e-commerce, and the logistics distribution is carried out by establishing a hierarchical logistics site. The current fitness value is calculated and the optimal individual is selected. Using the combination of direct logistics distribution and hierarchical logistics distribution, direct distribution is carried out for bulky goods and important distribution customers and hierarchical logistics distribution is used for customers in intensive logistics distribution destinations. According to the fitness value, the optimal individual of the newly generated population is selected, through the improvement of the whale position update method in the algorithm. The direct distribution method is mostly used in the logistics business where the journey is short, the distribution point is fixed, and there are many goods delivered at one time. The logistics enterprise does not need to store and distribute the goods. After the logistics enterprise obtains the goods from the supplier, it will be delivered directly to the customer, and in this way, the construction and operation costs of logistics sites are reduced, and it is suitable for logistics distribution under specific conditions. However, with the increase of modern logistics business demand, the distribution demand has become scattered and fragmented and most logistics enterprises no longer regard the direct logistics distribution method as the only distribution method of the enterprise but use it in combination with other distribution methods, as shown in Figure 1.

### 2.2. Hierarchical Distribution Network

Hierarchical logistics distribution is divided into two logistics methods: for small and medium-sized cities, a two-layer logistics distribution network is established that includes a combination of a general distribution site and several regional distribution sites. When it is delivered to the customer by the regional distribution site and when returning the goods, the goods first enter the regional logistics site, and then the regional logistics site is merged into the general distribution site. For large cities, because there are too many logistics orders, a total distribution site is not enough to complete the distribution and collection of a large number of orders, so an intermediate distribution site will be built between the first and second level distribution sites to assist in the management of logistics, forming a three-level city logistics and distribution network. The transit station means that it is used in the distribution network of large cities, and the distribution network of small and medium-sized cities does not use intermediate distribution stations, as shown in Figure 2.

## 3. Whale Optimization Algorithm

### 3.1. BWOA [16–20]

Reactive power scheduling optimization,

(1) $$\begin{array}{c} \min p=\min\sum_{i\in X}L_{i}*M_{i}. \end{array}$$

Short-term load forecasting,

(2) $$\begin{array}{c} x=\frac{\sum_{i\in X}L_{i}*M_{i}}{\sum_{i\in X}M_{i}}. \end{array}$$

Logistics and distribution calculation analysis selection,

(3) $$\begin{array}{c} \min F=\sum_{i=1}^{a}\sum_{j=1}^{b}x_{ij}c_{ij},\\ \min F=\sum_{i=1}^{n}\sum_{j=1}^{m}x_{ij}c_{ij}+\sum_{j=1}^{m}f_{j}. \end{array}$$

Surround prey,

(4) $$\begin{array}{c} \min F=\sum_{i=1}^{n}\sum_{j=1}^{m}x_{ij}c_{ij}+\sum_{j=1}^{m}\sum_{k=1}^{l}h_{jk}x_{jk}+\sum_{j=1}^{m}v_{j}{\left(w_{j}\right)}^{\sigma }. \end{array}$$

Bubble attack,

(5) $$\begin{array}{c} F=\sum_{i=1}^{k}\sum_{x=1}^{n}a_{xi}d\left(x,i\right)+\sum_{i=1}^{k}\sum_{j=1}^{m}b_{xi}d\left(i,j\right). \end{array}$$

Explore foraging,

(6) $$\begin{array}{c} W=\sum_{i=1}^{k}\left[\sum_{x=1}^{n}\max\left(g_{xi},\frac{v_{xi}}{60}\right)C\;d\left(x,i\right)\right]. \end{array}$$

Differential evolution algorithm,

(7) $$\begin{array}{c} \sum_{1}^{n}i\geq 1,\\ \sum_{1}^{n}\partial_{i}\leq 1. \end{array}$$

### 3.2. Rosenbrock [21–23]

(8) $$\begin{array}{c} \sum_{\theta =1}^{n}m_{\theta }\leq M. \end{array}$$

Single population development,

(9) $$\begin{array}{c} \left[\sum_{j=1}^{n}g_{ij},\sum_{x=1}^{n}g_{ij}\right]\geq 0,\\ d\left(x,i,j\right)\geq 0. \end{array}$$

Precocious astringent,

(10) $$\begin{array}{c} \left[\sum_{j\in D_{i}}j,\sum_{x\in D_{i}}x\right]\geq 1. \end{array}$$

High-dimensional space search,

(11) $$\begin{array}{c} F=\sum_{i=1}^{k}\sum_{x=1}^{n}a_{xi}d\left(x,i\right)+\sum_{i=1}^{k}\sum_{j=1}^{m}b_{xi}d\left(i,j\right)+\sum_{i=1}^{k}\sum_{j=1}^{m}t_{i}g_{i},\\ A=\left\{a_{1},a_{1},\ldots ,a_{i}\right\},\\ K_{1}=\left\{K1_{1},K2_{1},\ldots ,Kj_{1}\right\},\\ SSE_{1}={\sum_{m=1}^{j}\sum_{a_{m=1}\in Km_{1}}\left\|a_{m1}-Km_{1}\right\|}^{2}. \end{array}$$

#### 3.2.1. Quartic [24–26]

(12) $$\begin{array}{c} K_{2}=\left\{K1_{2},K2_{2},\ldots ,Kj_{2}\right\},\\ Kj_{2}=\text{mean}\left(a_{m1}\right). \end{array}$$

Global exploration capability,

(13) $$\begin{array}{c} SSE_{2}={\sum_{m=1}^{j}\sum_{a_{m=2}\in Km_{2}}\left\|a_{m2}-Km_{2}\right\|}^{2},\\ \Delta SSE_{2}=\left|SSE_{1}-SSE_{2}\right|. \end{array}$$

Local optimum,

(14) $$\begin{array}{c} \Delta SSE_{2}\leq \delta . \end{array}$$

Species diversity,

(15) $$\begin{array}{c} x\left(t+1\right)=x_{\text{best}}\left(t\right)+D*e^{bl}. \end{array}$$

Differential evolution algorithm,

(16) $$\begin{array}{c} x\left(t+1\right)=x_{\text{rand}}\left(t\right)-A*C*x_{\text{rand}}\left(t\right)-x\left(t\right). \end{array}$$

The overall coordination and balance of the logistics system are as follows:

(17) $$\begin{array}{c} p=\frac{\left|E_{x}-x\right|}{E_{x}},\\ x_{i}^{0}=\left(a_{i}-b_{i}\right)z_{i}+b_{i}. \end{array}$$

## 4. Simulation Experiment

### 4.1. Individual Elimination Strategy

When the WOA searches immediately, it moves closer to a random position. Although this method can ensure the diversity of the population to a certain extent, it is easy to produce inferior solutions that deviate from the optimal direction, which affects the convergence speed. In the cross selection strategy of the genetic algorithm, after each iteration, the population is sorted according to fitness and equally divided into two parts, one part is relatively high-quality individuals and the other part is relatively inferior individuals, and the two parts are subjected to pairwise arithmetic crossover to generate a new one. The population of, where S-LO = 111, S-LA = 107, C-LO = 54, C-LO = 62, WT = 44, and VO = 10. A crossover between high-quality individuals and low-quality individuals can ensure the diversity of the population. The original population is merged, and the new population, sorted by fitness, eliminates inferior individuals in the merged population and lets the retained high-quality individuals enter the next iteration, and S-LO = 110, S-LA = 94, C-LO = 86, C-LO = 75, WT = 46, and Vo = 3. S-LA guarantees the high quality of the population. Chaos S-LO mapping can be used to generate chaotic sequences, and C-LO has a better effect than pseudorandom numbers in generating WT chaotic sequences in population initialization as shown in Table 1 and Figure 3.

### 4.2. Partial Development Stage

The chaotic sequence is added on the basis of secondary reverse learning. The more commonly used discrete chaotic maps are Tent chaotic map and logistic chaotic map, and Ka = 4.08, Ao = 4.47, Io = 4.22, IT = 4.04, To = 4.52, No = 4.47, and *β* = 4.98. It is proved that the Tent chaotic map has better uniform traversal properties than the logistic chaotic map. If the current optimum is close to the local optimum, then a small step search pattern around the local optimum will trap the algorithm in a local extremum, and Io = 4.44, IT = 4.78, To = 4.39, No = 4.97, and *β* = 4. It is difficult to get rid of the shackles of local extrema. The introduction of Ka adaptive inertial weights is a good complement to optimize the limitations of the Ao whale algorithm. In the local development stage, Ka = 4.68 and Ao = 4.97; an effective mutation strategy makes it difficult for the whale population to get rid of the shackles of local optimum. See Table 2 and Figure 4.

### 4.3. Levy Flight Strategy

Levy flight is a kind of random walk (Randomly walk) motion of living organisms; bats, fruit flies, cuckoos, people, lights, etc., all have this levy flight behavior. The inertia weight plays an excellent role in balancing the global exploration ability and optimization performance of the intelligent algorithm, and HED = 3.82, ND = 3.58, HDE = 3.45, DIR = 3.66, DIT = 5.51, LAD = 4.7, *W* = 2.63, and KVAR = 2.16 is used in a variety of algorithms. The walking performance of this mechanism is a combination of the long-term short-distance search of HED and the occasional long-distance jump of KVAR, which is characterized by directional variability. The mutation strategy in the differential evolution algorithm is to randomly select two different individuals in the population, and HDE scales the vector difference and then performs vector synthesis with the individual to be mutated. See Table 3 and Figures 5 and6.

### 4.4. Improvement Strategies

The whale optimization algorithm simulates the unique bubble network attack mechanism of humpback whales. By calculating the fitness value of all search agents, the current optimal solution is selected, and then the circular contraction mechanism and the spiral up mechanism are selected. By calculating the fitness value of each whale, the optimal whale position bestX and its corresponding global optimal fitness value best f are found. When the population is initialized, the method of stochastic differential mutation is used in the particle swarm algorithm and the gray wolf algorithm, respectively. test function = 0.4, algorithm = 0.43, optimal = 0.49, average = 0.26, worst = 0.3, encircled prey in whale algorithm ND = 3.46, bubble attack HED = 3.34, exploration and foraging stage HDE = 3.64, compare current whale individuals, the fitness value LAD = 1.24, and the individual fitness value of the leading whale is DIT = 5.47. DIR = 3.43, *W* = 5.06, and KVAR = 1.77 to update the leading value and leading position and record the current global optimum value and optimum position at the same time. The selection of the circular contraction mechanism and the spiral up mechanism is performed (Figure 7).

As a meta-heuristic algorithm based on swarm intelligence, the WOA algorithm is the same as other meta-heuristic algorithms and has the advantages of fewer control parameters, simple implementation, and high flexibility. (1) Sphere has few control parameters: test function = 0.6, algorithm = 0.03, optimal = 0.63, average = 0.84, and worst = 0.49. The WOA algorithm mainly simulates the predation behavior of humpback whales and searches for the optimal solution by encircling the prey, searching for the prey, and attacking the bubble net. During the whole process, only two internal parameters A and C are utilized for the control of the exploration and development process. (2) BWOA is simple to implement, test function = 0.35, worst = 0.03, WOA algorithm obtains the optimal solution through algorithm = 0.35, optimal = 0.6 spiral equation, and iterative average = 0.37 position. (3) The flexibility of Rosenbrock is high optimal = 0.82. The implementation process of the WOA algorithm is simple, test function = 0.29, algorithm = 0.73, few parameters, and simple expressions. Practical problems in various fields can be solved by transforming or integrating other algorithms. Average = 0.11, worst = 0.5, which has the characteristics of high flexibility. See Table 4 and Figure 8.

## 5. Conclusion

As a meta-heuristic algorithm based on swarm intelligence, the WOA algorithm has few control parameters and searches for the optimal solution by encircling the prey, searching for the prey, and attacking the bubble net. BWOA is simple to implement. In the process of algorithm execution, the initial population, global exploration, and local development stages have shortcomings. Therefore, it is necessary to optimize the WOA algorithm.

Based on WOA, this study conducts a high-performance computing analysis and location selection of logistics distribution center space. It is obtained: 1. Using the combination of direct logistics distribution and hierarchical logistics distribution, the two parts perform pairwise arithmetic crossover to generate a new population, where S-LO = 111, S-LA = 107, C-LO = 54, C-LO = 62, WT = 44, and Vo = 10. A crossover between high-quality individuals and low-quality individuals can ensure the diversity of the population. The original population and the new population are merged, sorted by fitness, eliminate inferior individuals in the merged population and let the retained high-quality individuals enter the next iteration, and S-LO = 110, S-LA = 94, C-LO = 86, C-LO = 75, WT = 46, and Vo = 3. S-LA guarantees the high quality of the population. 2. The logistic chaos map Ka = 4.08, Ao = 4.47, and Io = 4.22. Tent chaotic map has better uniform traversal properties IT = 4.04, To = 4.52, N-o = 4.47, and *β* = 4.98 than the logistic chaotic map. If the current optimum is close to the local optimum, the small-step search pattern around the local optimum will cause the algorithm to fall into the local extremum, and Io = 4.44, IT = 4.78, To = 4.39, No = 4.97, and *β* = 4, get rid of local extrema bound. 3. The concept of random difference variation is used in the particle swarm algorithm and gray wolf algorithm, respectively. test function = 0.4, algorithm = 0.43, optimal = 0.49, average = 0.26, worst = 0.3, encircled prey in whale algorithm ND = 3.46, bubble attack HED = 3.34, exploration and foraging stage HDE = 3.64, comparing current whale individuals the fitness value LAD = 1.24, and the individual fitness value of the leading whale is DIT = 5.47. DIR = 3.43, *W* = 5.06, and KVAR = 1.77 to update the leading value and leading position and record the current global optimum value and optimum position at the same time. 4. Sphere has few control parameters: test function = 0.6, algorithm = 0.03, optimal = 0.63, average = 0.84, and worst = 0.49. The WOA algorithm mainly simulates the predation behavior of humpback whales and searches for the optimal solution by encircling the prey, searching for the prey, and attacking the bubble net. During the whole process, only two internal parameters A and C are utilized for the control of the exploration and development process. BWOA is simple to implement, test function = 0.35, worst = 0.03, WOA algorithm obtains the optimal solution through algorithm = 0.35, optimal = 0.6 spiral equation, and iterative average = 0.37 position. Rosenbrock flexibility is high optimal = 0.82. The implementation process of the WOA algorithm is simple, test function = 0.29, algorithm = 0.73, few parameters, and simple expressions. Practical problems in various fields can be solved by transforming or integrating other algorithms. Average = 0.11 and worst = 0.5, which has the characteristics of high flexibility. [27].

## Figures and Tables

**Figure 1:** Enterprise logistics network.

**Figure 2:** Logistics optimization distribution network.

**Figure 3:** Individual elimination strategy parameters.

**Figure 4:** Local development parameter settings.

**Figure 5:** Levy flight strategy.

**Figure 6:** Flight node parameters.

**Figure 7:** Whale optimization algorithm.

**Figure 8:** Algorithm comparison.

**Table 1:** Parameters of individual elimination strategy.

S-LO	S-LA	C-LO	C-LO	WT	Vo
99	116	78	77	28	3
119	102	62	56	27	9
90	111	74	71	20	9
96	111	68	60	28	9
110	94	86	75	46	3
94	107	72	65	22	9
99	96	67	54	42	8
114	102	73	90	31	10
92	109	63	81	40	8
105	117	90	65	48	9
111	107	54	62	44	10

**Table 2:** Local development parameter settings.

Parameter	Ka	Ao	Io	IT	To	N-o	*β*
Ka	4.08	4.68	4.46	4.89	4.63	4.08	4.83
Ao	4.13	4.97	4.87	4.01	4.53	4.47	4.77
Io	4.40	4.44	4.39	4.88	4.62	4.22	4.35
IT	4.27	4.78	4.69	4.13	4.77	4.04	4.33
To	4.21	4.39	4.46	4.58	4.43	4.52	4.53
N-o	4.00	4.97	4.94	4.21	4.12	4.47	4.93
Β	4.08	4.00	4.01	4.53	4.13	4.98	4.90

**Table 3:** Flight node parameters.

HED	ND	HDE	DIR	DIT	LAD	W	KVAR
3.41	3.30	3.85	3.16	3.74	3.90	1.59	2.65
3.65	3.73	3.55	3.49	3.19	1.09	1.67	1.25
3.14	3.16	3.84	3.76	1.39	3.73	4.80	2.00
3.82	3.58	3.45	3.66	5.51	4.70	2.63	2.16
3.34	3.46	3.64	3.43	5.47	1.24	5.06	1.77
3.50	3.87	3.31	3.93	2.97	4.42	4.86	3.78
3.34	3.98	3.44	3.41	3.08	2.46	1.64	5.21
3.53	3.85	3.00	3.86	1.17	3.70	4.59	1.02

**Table 4:** Comparison of algorithms.

	Test function	Algorithm	Optimal	Average	Worst
Sphere	0.60	0.03	0.63	0.84	0.49
BWOA	0.40	0.43	0.49	0.26	0.30
Rosenbrock	0.10	0.35	0.18	0.53	0.04
Quartic	0.35	0.35	0.60	0.37	0.03
Ackley	0.29	0.73	0.82	0.11	0.50
Schwefel's	0.89	0.77	0.14	0.81	0.47

## Data Availability

The experimental data used to support the findings of this study are available from the corresponding author upon request.
